# Computer Intelligent Algorithm in the Recovery of the Elbow Joint Sports Injury Model

**DOI:** 10.1155/2022/5044952

**Published:** 2022-01-04

**Authors:** Huiyu Duan, Shenglong Xun, Yichen Bao, Gong Zhang

**Affiliations:** ^1^Department of Physical Education, Inner Mongolia University of Technology, Hohhot 010051, China; ^2^School of Physical Education, Liaoning Normal University, Dalian 116029, China; ^3^Institute of Foreign Language, Inner Mongolia University of Technology, Hohhot 010051, China

## Abstract

In this study, the inverse kinematics mathematics computer intelligent algorithm model is used to study the sports injuries of the elbow joint of adolescents. At the same time, we simulated the movement parameter changes during the rehabilitation training of the patient's wrist and proposed a joint angular velocity function based on cubic fitting. Research has found that when the training scene changes greatly or the target task is changed, the smoothness of the elbow joint movement will change. The research conclusions of this article provide a theoretical basis for the selection of man-machine action points and the formulation of rehabilitation training methods. This article establishes the degree-of-freedom simulation model of the operating arm, which is the number of independent position variables in the operating arm, and these position variables determine the positions of all parts in the mechanism.

## 1. Introduction

The pneumatic artificial muscle (PAM) has flexible characteristics. Compared with the traditional pneumatic actuator, it has the advantages of simple structure, large output force-to-weight ratio, high energy conversion efficiency, and good bionic performance. We use it as the driver of the human-like robotic arm to reduce the cost and improve the flexibility of the mechanism [1]. At present, the structure of pneumatic muscle bionic manipulators is continuously researched and developed at home and abroad, and many eye-catching results have been obtained.

Establishing an accurate kinematics model of the mechanism is the primary issue in the research process of the bionic manipulator structure. It is the basis and guarantees for mechanism mechanics, error, and control research and analysis. Pneumatic muscle bionic manipulator is a flexible mechanism [2]. Among them, the finite element method is difficult to be an effective method for the kinematics analysis of flexible mechanisms due to the harsh requirements of the initial conditions. The geometric analysis method mainly aims at the fully flexible mechanism with distributed flexibility, but the method currently does not have a unified procedure. It can only determine the appropriate algorithm based on the specific structure and is not universal. It has great disadvantages for fully flexible mechanisms with distributed flexibility.

This study established a three-degree-of-freedom pneumatic muscle bionic elbow joint to establish its pseudorigid body model [3]. Second, according to the established equations, the simulation analysis of the changes of the pneumatic muscle length is under different motion trajectory conditions [4]. Finally, a virtual prototype of the mechanism is constructed based on the pseudorigid body model, and a simulation system model of the pneumatic muscle bionic elbow joint is built. This verifies the accuracy of the built kinematics inverse solution model.

## 2. Organization Description

The bionic elbow joint comprises of forearm disc 1, upper arm disc 2, Hooke hinge 3, pneumatic muscle 4, and support rod 5 (Figure 1). One of the Hooke hinges is placed at the centre point of the forearm disc [5]. The rest are placed on the forearm disc and the upper arm disc according to the equilateral triangle inscribed in the disc. The three pneumatic muscles are connected to the forearm disc and the upper arm disc through the Hooke hinge, and there is an axial rotation between the Hooke hinges. The upper end of the support rod is connected with the centre point of the forearm disc through the Hooke hinge, and there is an axial rotation between the Hooke hinges [6]. The lower end is fixedly connected with the centre point of the upper arm disc through a thread. The forearm disc can be rotated by driving 3 pneumatic muscles to control its internal pressure and flow rate.

## 3. Establishment of the Inverse Kinematics Equation of the Mechanism

Because the pneumatic muscle is a flexible part and the bionic elbow joint is a rigid-flexible hybrid mechanism, the “pseudorigid body model method” can be used to establish the kinematics equation of the pneumatic muscle bionic elbow joint. We regard the pneumatic muscle as a cylinder pair, which is composed of two components. Since the support rod and the upper arm disc are firmly connected, they are regarded as components [7].

(1) $$\begin{array}{c} F=6\left(n-g-1\right)+\sum_{i=1}^{g}f_{i}=6\left(8010-1\right)+2\times 7+2\times 3+1=3. \end{array}$$

First, establish a fixed coordinate system *O*_*B*_ − *X*_*B*_, *Y*_*B*_, *Z*_*B*_ at the centre point of the upper arm disc. The *X*_*B*_ axis passes through the hinge point *B*_3_. Then, establish the moving coordinate system *O*_*p*_ − *X*_*p*_, *Y*_*p*_, *Z*_*p*_ at the centre point of the forearm disc. Its *X*_*p*_ axis passes through the hinge point *b*_3_. *Y*_*p*_ of the forearm platform [8]. The axis intersects the side *b*_1_*b*_3_ and is parallel to the side *b*_1_*b*_2_. We take the fixed coordinate system *O*_*B*_ − *X*_*B*_, *Y*_*B*_, *Z*_*B*_ as the reference coordinate system. We assume that the rotation sequence of the mechanism is *Z*_*p*_ − *Y*_*p*_ − *X*_*p*_.

(2) $$\begin{array}{c} R=R_{Z_{p}}\left(\varphi \right)R_{Y_{p}}\left(\theta \right)=\left(\begin{array}{ccc} \cos\;\varphi & -\sin\;\varphi & 0\\ \sin\;\varphi & \cos\;\varphi & 0\\ 0 & 0 & 1 \end{array}\right)\left(\begin{array}{ccc} \cos\;\theta & 0 & \sin\;\theta \\ 0 & 1 & 0\\ -\sin\;\theta & 0 & \cos\;\theta \end{array}\right). \end{array}$$

We describe the rotation matrix of equation (2) as

(3) $$\begin{array}{c} R=\left(\begin{array}{ccc} x_{1} & x_{m} & x_{n}\\ y_{1} & y_{m} & y_{n}\\ z_{1} & z_{m} & z_{n} \end{array}\right). \end{array}$$

Then, the link vector between the corresponding hinge points of the two discs is

(4) $$\begin{array}{c} l_{i}e_{i}=P+Rb_{i}-B_{i}. \end{array}$$

If we substitute the coordinates of Hooke's hinge *b*_*i*_, *B*_*i*_ into equation (3) and take the vector modulus, there is a scalar equation for the rod length [9]. After we expand the square of formula (4) and eliminate *e*_*i*_, the length of each pneumatic muscle can be obtained as

(5) $$\begin{array}{c} l_{i}^{2}=B_{ix}^{2}+B_{iy}^{2}+b_{ix}^{2}\left(x_{l}^{2}+y_{l}^{2}+z_{l}^{2}\right)+b_{iy}^{2}\left(x_{m}^{2}+y_{m}^{2}+z_{m}^{2}\right)\\ +2b_{ix}b_{iy}\left(x_{l}x_{m}+y_{l}y_{m}+z_{l}z_{m}\right)-2B_{ix}\left(b_{ix}x_{l}+b_{iy}x_{m}\right)\\ -2B_{iy}\left(b_{ix}y_{l}+b_{iy}y_{m}\right)+2b_{ix}zz_{l}+2b_{iy}zz_{m}+z^{2}. \end{array}$$

According to the orthogonality *RR*^*T*^=*E* of the rotation matrix, equation (5) can be reduced to

(6) $$\begin{array}{c} l_{i}^{2}=B_{ix}^{2}+B_{iy}^{2}+b_{ix}^{2}+b_{iy}^{2}-2B_{ix}\left(b_{ix}x_{l}+b_{iy}x_{m}\right)-2B_{iy}\left(b_{ix}y_{l}+b_{iy}y_{m}\right)\\ +2b_{ix}zz_{l}+2b_{iy}zz_{m}+z^{2}. \end{array}$$

If we substitute equations (3) and (4) into equation (6) and root the square, we can get three equations of pneumatic muscle length change as

(7) $$\begin{array}{c} \left\{\begin{array}{c} l_{1}=\sqrt{2r^{2}\left(1-x_{l}\right)+z\left(z+2rz_{l}\right)};\\ l_{2}=\sqrt{2r^{2}+z^{2}-\frac{r^{2}}{2}\left(x_{l}+\sqrt{3}x_{m}+\sqrt{3}y_{l}+3y_{m}+\frac{2\sqrt{3}}{r}zz_{m}+\frac{2}{r}zz_{l}\right)};\\ l_{3}=\sqrt{2r^{2}+z^{2}-\frac{r^{2}}{2}\left(x_{l}-\sqrt{3}x_{m}-\sqrt{3}y_{l}+3y_{m}-\frac{2\sqrt{3}}{r}zz_{m}+\frac{2}{r}zz_{l}\right).} \end{array}\right. \end{array}$$

Equation (7) is the inverse kinematics equation of the pneumatic muscle bionic elbow joint. We can obtain the inverse solution equation of the mechanism velocity by deriving the two ends of the equation group (8):

(8) $$\begin{array}{c} \upsilon_{l}=J^{-1}\upsilon_{p}, \end{array}$$

where *υ*_*l*_=(*υ*_*l*1_, *υ*_*l*2_, *υ*_*l*3_)^*T*^, and *υ*_*P*_=(*ω*_*ψ*_*r*, *ω*_*θ*_*r*, *ω*_*φ*_*r*)^*T*^*J*^−1^ is the coefficient matrix of *υ*_*p*_. This is also the inverse matrix of the Jacobian matrix of the institution. We can obtain the acceleration equation of the mechanism by deriving the two ends of equation (8) again:

(9) $$\begin{array}{c} a_{l}={\left(J^{-1}\right)}^{\prime }\upsilon_{P}+J^{-1}\upsilon_{p}^{\prime }, \end{array}$$

a numerical example of inverse kinematics solution.

We assume that the radius of the upper arm disc and the forearm disc of the mechanism are both 38.5 mm. The position coordinate of the origin of the moving coordinate system *O*_*p*_ − *X*_*p*_, *Y*_*p*_, *Z*_*p*_ relative to the fixed coordinate system *O*_*B*_ − *X*_*B*_, *Y*_*B*_, *Z*_*B*_ is *P*=(0,0,250)^*T*^ [10]. The result is shown in Figure 2.

When the front arm disc rotates relative to the *X*_*B*_ axis, the two pneumatic muscles that are symmetrical to the *X*_*B*_ axis also exhibit symmetry in length changes. The length of another pneumatic muscle that intersects perpendicularly to the *X*_*B*_ axis remains unchanged (Figure 2(a)). When the front arm disc rotates relative to the *Y*_*B*_ axis, the length change curve of the two pneumatic muscles symmetrical to the *X*_*B*_ axis is the same variable [11]. The other pneumatic muscle length change curve amplitude is larger than the other two, and the phase difference is 180° (Figure 2(b)). When the front arm disc rotates relative to the *Z*_*B*_ axis, the length change curves of the three pneumatic muscles are the same (Figure 2(c)). When the front arm disc moves in a circular motion, the phases of the length change curves of the three pneumatic muscles are 120° apart from each other (Figure 2(d)). It can be seen from Figure 3 that although the motion trajectories of the reference points are different, the changes in the length of the three pneumatic muscles are continuous and stable without sudden changes.

## 4. Verification of the Inverse Kinematics Equation

We need to verify further the accuracy of the pneumatic muscle bionic elbow joint inverse kinematics equation. We establish the virtual prototype of the joint mechanism and its simulation system model in MATLAB/Simulink according to the pseudorigid body model of the mechanism [12]. According to equation (9), the theoretical length is calculated. The difference between it and the actual length is used as the input of the PID controller. We get the trajectory curve of the forearm disc angle of the mechanism by adjusting the PID parameters. We compare it with the expected trajectory, and the result is shown in Figure 4.

It can be seen from Figure 4 that the forearm disc rotation angle trajectory curve coincides with the desired trajectory curve. The error changes are shown in Figures 4(b) and 4(d). This verifies the accuracy of the mathematical model of the inverse kinematics solution of the established mechanism.

## 5. Conclusion

We obtain the inverse kinematics solution equation of the mechanism according to the model. Second, we complete the numerical simulation analysis of the inverse kinematics solution of the mechanism according to the equations. According to the inverse kinematics equation, the PID control of the virtual prototype is implemented to verify the accuracy of the inverse equation. The trajectory curve of the forearm disc rotation angle of the bionic elbow joint of the pneumatic muscle has a higher degree of coincidence with the desired trajectory curve. In this way, verifying the accuracy of the inverse solution equation is realized, and the reliability of the simulation results is enhanced. This lays the foundation for the analysis of the mechanism's kinematics and mechanical properties.

## Figures and Tables

**Figure 1:** Pneumatic muscle bionic elbow joint model.

**Figure 2:** Pneumatic muscle length change curve. (a) *ψ*=50  sin(*t*). (b) *θ*=50  sin(*t*). (c) *φ*=20  sin(*t*). (d) *ψ*=30  sin(*t*), *θ*=30  cos(*t*).

**Figure 3:** Pneumatic muscle bionic elbow joint virtual prototype and simulation system model.

**Figure 4:** Control simulation results. (a) Tracking (*ψ*=*π*/9 · sin(*t*)). (b) Tracking error (*ψ*=*π*/9 · sin(*t*)). (c) Square wave signal track (*ψ*=*π*/36). (d) Square wave signal track error (*ψ*=*π*/36).

## Data Availability

The data used to support the findings of this study are available from the corresponding author upon request.
